# Fungal Skin Disease Classification Using the Convolutional Neural Network

**DOI:** 10.1155/2023/6370416

**Published:** 2023-05-30

**Authors:** Tsedenya Debebe Nigat, Tilahun Melak Sitote, Berihun Molla Gedefaw

**Affiliations:** ^1^Information Technology, Faculty of Computing and Informatics, Jimma Institute of Technology, Jimma University, Jimma, Oromia, Ethiopia; ^2^Department of Computer Science and Engineering (CSE), School of Electrical Engineering and Computing, Adama Science and Technology University (ASTU), P.O. Box 1888, Ethiopia; ^3^Health Informatics, College of Medicine and Health Science, Arbaminch University, P.O. Box 21, Arbaminch, Ethiopia

## Abstract

Skin is the outer cover of our body, which protects vital organs from harm. This important body part is often affected by a series of infections caused by fungus, bacteria, viruses, allergies, and dust. Millions of people suffer from skin diseases. It is one of the common causes of infection in sub-Saharan Africa. Skin disease can also be the cause of stigma and discrimination. Early and accurate diagnosis of skin disease can be vital for effective treatment. Laser and photonics-based technologies are used for the diagnosis of skin disease. These technologies are expensive and not affordable, especially for resource-limited countries like Ethiopia. Hence, image-based methods can be effective in reducing cost and time. There are previous studies on image-based diagnosis for skin disease. However, there are few scientific studies on tinea pedis and tinea corporis. In this study, the convolution neural network (CNN) has been used to classify fungal skin disease. The classification was carried out on the four most common fungal skin diseases: tinea pedis, tinea capitis, tinea corporis, and tinea unguium. The dataset consisted of a total of 407 fungal skin lesions collected from Dr. Gerbi Medium Clinic, Jimma, Ethiopia. Normalization of image size, conversion of RGB to grayscale, and balancing the intensity of the image have been carried out. Images were normalized to three sizes: 120 × 120, 150 × 150, and 224 × 224. Then, augmentation was applied. The developed model classified the four common fungal skin diseases with 93.3% accuracy. Comparisons were made with similar CNN architectures: MobileNetV2 and ResNet 50, and the proposed model was superior to both. This study may be an important addition to the very limited work on the detection of fungal skin disease. It can be used to build an automated image-based screening system for dermatology at an initial stage.

## 1. Introduction

Skin is the outermost layer spread throughout the body, accounting for 16% of the body mass [1]. It is the first line of defense to protect the vital organs of our body from harm. It is necessary to give proper attention to the overall health of the skin. Changes in its normal functioning can affect other parts of the body. Any disorder that affects the skin is a skin disease. Skin is often affected by diseases caused by fungus, bacteria, viruses, allergies, and dust. There are more than 3000 known skin diseases worldwide [2]. Skin disease is one of the major global health issues across all age groups that affects about 900 million people [2, 3]. It is the fourth leading cause of skin related illness [4]. It is a significant cause of infection in sub-Saharan Africa [5]. An estimated 21–87% of children in Africa are affected by skin disease [6]. According to the WHO report of 2018, skin disease-related deaths in Ethiopia reached 2,459, accounting for 0.40% of total deaths [7]. The most common skin illnesses include eczema, melanoma, vitiligo, mycosis, papillomas, impetigo, scabies, herpes, dermatitis, warts, psoriasis, acne, tinea corporis, tinea pedis, and tinea capitis [8]. If not detected and treated promptly, they are dangerous and can spread easily. The disability caused by diseases can have a psychological impact on people that affects their education, relationships, self-esteem, career choices, and social, sexual, and leisure activities. This can also lead to depression, frustration, isolation, and even suicide [9, 10].

Fungal skin disease is one of the most common types of skin disease. Superficial fungal infections affect the hair, nails, epidermis, and mucosa. Dermatophytes are the most common cause of superficial fungal infections. It is prevalent in developing nations. Tinea corporis, tinea capitis, tinea pedis, tinea cruises, and pityriasis vesicular are the most common fungal infections [11]. Tinea corporis is more prevalent in children and young adults and infects the whole body. Tinea capitis infects the skin around the scalp. Tinea pedis generally infects the leg and foot, beginning between the toes. It is common in people who have sweaty feet while wearing tight-fitting shoes. Tinea unguium, or onychomycosis, is a fungal skin disease that infects the nail. The global prevalence of onychomycosis is 5.5% and contributes 50% to all nail diseases [12]. Tinea infections can be difficult to diagnose and treat accurately because of the similarity between different types of fungal morphology. As a result, image-based approaches to detection and diagnosis of fungal skin diseases may be effective. Early detection and diagnosis of fungal skin disease are critical to providing appropriate treatment and preventing further spread. Fever, pain, and dyspnea are some of the clinical symptoms of fungal skin diseases. These symptoms are not specific to fungal skin diseases, and the fungal spore microscopic image of the fungal spores is complex, making early detection and diagnosis difficult [13]. Common methods for the diagnosis of fungal skin diseases are based on blood tests, history, symptom analysis, skin scraping, visual inspection, dermoscopy, and skin biopsy. These diagnosis methods are time-consuming, require an extensive understanding of the domain, and are vulnerable to subjective errors.

Detection, diagnosis, and classification of skin disease were carried out previously by different studies. They have used different methodologies, and therefore, the performances of the models are different. Velasco et al. proposed smartphone-based skin disease detection. Their system recognized acne, eczema, pityriasis rosea, psoriasis, tinea corporis, varicella (chickenpox), and vitiligo with an accuracy of 94% [14]. Wu et al. compared five pretrained deep learning frameworks for the diagnosis of six facial skin conditions from a clinical image and using an InceptionResNet_V2 [15]. The reported precision of their model has been 77% [15]. Kamulegeya et al. developed a skin disease identification model of Uganda [16]. They have used a black-color image dataset. The accuracy was low (17%). They concluded that the model is poor for detecting fungal infections like tinea. In all previous scientific works, highly prevalent skin fungal diseases such as tinea capitis, tinea pedis, and tinea unguium were not significantly considered. In this study, we used CNN to classify the most common fungal skin diseases.

This study may be an important contribution to the classification of fungal skin diseases, where there are few previous scientific works, especially on high-burden diseases such as tinea pedis and tinea corporis. The performance of the proposed model is superior to models with similar architecture. More importantly, it can be very helpful in the early identification of the most common fungal skin diseases by building an automated screening system. It can be integrated with knowledge-based systems and clinical decision support systems to support practitioners. This will be useful, especially for resource-limited health facilities that have an acute shortage of diagnostic tools and means. Timely diagnosis and effective medication can be achieved with these systems.

The remainder of the paper has been organized into three sections. In Section 2, the materials and method used in the study to classify the most common fungal skin diseases have been discussed. Details of the dataset, preprocessing techniques, augmentation, modeling, and evaluation have been described. In Section 3, experiments, results, discussion, and evaluations of the proposed method are incorporated. The conclusion that highlights the main findings and inferences has been incorporated in Section 4.

## 2. Materials and Method

The aim of this study was to effectively classify the most common fungal skin diseases, tinea pedis, tinea capitis, tinea corporis, and tinea unguium, using CNN. As shown in the work flow diagram in Figure 1, it was carried out in a series of steps that included preparation of the dataset, preprocessing, image annotation, modeling, and evaluation.

### 2.1. Dataset

The dataset for this study was collected from the Dr. Gerbi Medium Clinic in Jimma, Ethiopia. The images were captured after the diagnosis was confirmed by a dermatologist. Tinea pedis, tinea capitis, Tinea Corporis, and tinea unguium were the four labels in the collected images. The dataset comprises a total of 407 images of the selected four fungal skin diseases.  Table 1 displays the distribution and percentages.

### 2.2. Image Preprocessing

Image preprocessing is a technique to improve the quality of images by applying different techniques. Most original medical images contain irrelevant parts that require preprocessing. Image preprocessing techniques are used ahead of classification to remove such irrelevant parts of the images, with the goal of improving image visualization and model performance [17]. Normalization, image color conversion, and image resizing were specific techniques used in this study. The original images were not uniform in size, and they were resized into 120 × 120, 150 × 150, and 224 × 224 pixels. After the size of all acquired images became uniform, the color was converted from RGB to grayscale. Feature extraction is a technique that changes the original features of the data into a new, smaller set of features that is more informative. This smaller set of informative features is critical for recognition to distinguish between different labels. CNN is effective in the extraction of deep features. The powerful learning ability of deep CNN is primarily due to the use of multiple feature extraction stages that can automatically learn representations from the data [18].

### 2.3. Augmentation

Data augmentation is a technique that is used to artificially increase the size of the dataset. It is one way to prevent deep learning models from overfitting. There are several data augmentation techniques, such as cropping, rotations, flipping, translations, contrast adjustment, and scaling. In this study, we augment 407 images labeled into four classes: tinea capitis, tinea corporis, tinea pedis, and tinea unguium. After augmentation, we have a dataset of 1069 images, as shown in Table 2.

### 2.4. Modeling and Evaluation

The deep learning model proposed for this study is CNN. It is one of the implementations of a neural network that has been widely used in image-based learning. Automatic extraction and selection of features are two of the main strengths of deep learning models [19]. CNN in particular is effective in extracting deep features. It has been suggested that the accuracy of disease detection can be greatly enhanced with the combination of clinical and imaging data and the use of newer artificial intelligence methods such as deep learning [20]. Deep learning has been used effectively in medical image detection and classification [21–23]. To identify patients with COVID-19 in their early stages of the disease, NASNet, a state-of-the-art pretrained convolutional neural network for image feature extraction, has been used effectively [21]. In the study, COVID-19 cases were identified without misclassification errors. Similarly, eight well-known CNN models were used for feature extraction in the detection of B-ALL lymphoblasts [22]. Early detection of diseases is usually vital for effective and timely intervention [23, 24]. With current medical devices and technology, early detection or identification is getting better, but people may not reach to diagnosis centers in time or are too expensive for some, especially in developing countries [25]. The symptoms and signs of some of the diseases are too similar and asymmetric for extremely large areas, making identification difficult [26]. We believe that the proposed CNN model is appropriate for the classification of fungal skin diseases. In order to evaluate the performance, commonly applied evaluation metrics such as accuracy, precision, recall, and *f*1-score have been used, as shown in the following equations:

(1) $$\begin{array}{c} accuracy=\frac{TP+TN}{TP+TN+FP+FN}\text{,}\\ precision=\frac{TP}{TP+FP}\text{,}\\ \begin{array}{c} recall=\frac{TP}{TP+FN},\\ f1-score=2*\frac{precision*recall}{precision+recall},\\ sensitivity=\frac{TP}{TP+FP},\\ specificity=\frac{TN}{TN+FN}, \end{array} \end{array}$$

where TP is true positive, FP is false positive, TN is true negative, and FN is false negative.

## 3. Results and Discussion

Reducing the image to its optimal size decreases processing time and cost. The dataset consists of images of different sizes. We resized images to the sizes of 120 × 120, 150 × 150, and 224 × 224. We carried out modeling by varying image sizes to obtain optimal performance. As the size of the image increases, it needs more computational time. The maximum accuracy obtained was with an image size of 224 × 224. These experiments have been discussed as follows: The first was carried out with an image size of 120 × 120. The training accuracy of the model has been 85% and its validation accuracy has been 81%, as shown in Figure 2.

Then, modeling was carried out with an image size of 150 × 150. The training accuracy of the model has increased to 86% and its validation accuracy to 83%, as shown in Figure 3.

Lastly, modeling was carried out with an image size of 224 × 224. The training accuracy of the model has increased to 93.3% and its validation accuracy to 87.3%. The result showed that modeling with an image size of 224 × 224 has the best performance when compared with modeling with image sizes of 120 × 120 and 150 × 150, even if it is computationally more expensive. The accuracy and loss are shown in Figure 4.

The modeling confusion matrix with an image size of 224 × 224 is shown in Figure 5. From the total of 214 validation images, 187 have been correctly classified and 27 incorrectly classified. As shown in Table 3, the performance of the model is an accuracy of 93.3%, a sensitivity of 86.4%, a specificity of 95.4%, a precision of 87.3%, a recall of 86.4%, and an *F*1 score of 86.8%.

Hyperparameter optimization is an important task to obtain optimal performance. We have conducted modeling with two activation functions, ReLU and ELU, separately to obtain optimal performance. The image size was 224 × 224, and the color mode was RGB. Firstly, the model was trained using a 224 × 224 image size in the RGB color mode with an ELU activation function. The training accuracy of the model is 88.5% and its validation accuracy is 81%, as shown in Figure 6.

The model was trained using 224 × 224 pixels of image size, RGB color images, and ReLU as an activation function. The training accuracy of the model has been 93.3%, and its validation accuracy has been 87.3%. This result shows that use of the ReLU activation function enhanced the performance. We conducted two modeling experiments using RGB and grayscale color modes with an image size of 224 × 224 for the classification of fungal skin diseases in order to identify an appropriate color mode. The training accuracy of the model has been 76.0%, and its validation accuracy has been 65.0%. The result showed that the classification accuracy of using RGB colors is better than using grayscale color modes. The training/validation accuracy and loss using RGB color are shown in Figure 7.

A comparison has been made with similar CNN architectures using the same dataset and parameters. There are different types of deep neural network models, such as AlexNet, ResNet, MobileNet, VGG16, VGG19, and GoogleNet. From these models, we have selected MobileNetV2 and ResNet50 to compare the proposed model. The MobileNetV2 model was trained using the 224 × 224 image size, the RGB color channel, and the ReLU activation function. The training accuracy of the model has been 90.5% and its validation accuracy has been 81.0%, as shown in Figure 8. This means that HSFDCModel outperformed MobileNet V2.

Similarly, the ResNet 50 model was trained using the 224 × 224 image size, RGB color channel, and ReLU activation function. The training accuracy of the model has been 89% and its validation accuracy has been 86%, as shown in Figure 9. This means that HSFDCModel also outperformed ResNet50.

In general, we conducted four different experiments to achieve optimal performance and validated them through comparison. These experiments were carried out to find an appropriate image size, activation function, and color channel. The optimal result has been obtained with an image size of 224 × 224, the ReLU activation function, and the RGB color channel. The comparison with similar CNN architectures, MobileNetV2 and ResNet50, showed that the proposed CNN model significantly outperformed both of them. The stated results have been shown in Table 4 and Figure 10.

## 4. Conclusions

Millions of people around the world have been affected by skin diseases. It is one of the common causes of infection in resource-limited regions like sub-Saharan Africa. Early detection and intervention are important to minimize its impact. However, existing state-of-the-art diagnostic techniques such as laser and photonics-based technologies are not affordable for resource-limited nations. This makes image-based methods more effective. There have been studies to detect and classify skin diseases using different deep learning techniques. However, only few of them focused on highly prevalent fungal skin diseases such as tinea pedis and tinea corporis. In this study, CNN has been used to classify four common fungal skin diseases: tinea capitis, tinea pedis, tinea corporis, and tinea unguium. Different experiments were carried out to obtain the optimum performance. An accuracy of 93.3% has been obtained with an image size of 224 × 224, ReLU activation function, and RGB color channel. Comparisons were made with two similar CNN architectures: MobileNetV2 and ResNet 50. The proposed CNN model significantly outperformed both of them. This study may be helpful in the early identification of the four common fungal skin diseases in health facilities that have an acute shortage of skin disease diagnosis equipment. This can be important for timely treatment. An image-based automated fungal skin disease screening system can also be built. To improve performance and scalability, the study can be extended in the future by increasing the number of datasets, the number of fungal skin diseases to be classified, and experimenting with hybrid deep learning techniques. Knowledge-based systems and clinical decision support systems can also be developed from the study.

## Figures and Tables

**Figure 1:** Work flow diagram.

**Figure 2:** Training/validation accuracy and loss for image size of 120 × 120.

**Figure 3:** Training/validation accuracy and loss for image size of 150 × 150.

**Figure 4:** Accuracy and loss for 224 × 224 image size.

**Figure 5:** Confusion matrix of HFSDM for 224 × 224 image size.

**Figure 6:** Training/validation accuracy and loss with ELU activation.

**Figure 7:** Training/validation accuracy and loss using grayscale color.

**Figure 8:** Training/validation accuracy and loss of MobileNet V2.

**Figure 9:** Training/validation accuracy and loss of ResNet50.

**Figure 10:** Sample classification of fungal skin disease.

**Table 1:** Dataset.

Fungal skin diseases	No. of images	Percentage (%)
Tinea capitis	120	29.5
Tinea pedis	96	23.6
Tinea corporis	71	17.4
Tinea unguium	120	29.5
Total number of images	407	100

**Table 2:** Dataset after augumentation.

Fungal skin diseases	No. of images before augmentation	No. of images after augmentation
Tinea capitis	120	304
Tinea pedis	96	264
Tinea corporis	71	229
Tinea unguium	120	272
Total number of images	407	1069

**Table 3:** HSFDCModel evaluation result.

Metrics	Values (%)
Accuracy	93.3
Sensitivity/recall	86.4
Specificity	95.4
Precision	87.3
*F*1 score	86.8

**Table 4:** Summary of the experimental result.

Models	Image sizes	Activation functions	Color channels	Training accuracy (%)	Validation accuracy (%)
HSFDCM	120 × 120	ReLU	RGB	85.0	81.0
HSFDCM	150 × 150	ReLU	RGB	86.0	83.0
HSFDCM	224 × 224	ReLU	RGB	93.3	87.3
HSFDCM	224 × 224	ELU	RGB	88.5	81.0
HSFDCM	224 × 224	ReLU	Gray	76.0	65.0
MobileNetV2	224 × 224	ReLU	RGB	90.5	81.0
ResNet50	224 × 224	ReLU	RGB	89.0	86.0

## Data Availability

The data used to support the findings of this study are available upon request to the corresponding author.
